# Analysis of Eastern Asia’s Contributions to Major Orthopaedic Journals in the Past 21 Years

**DOI:** 10.7759/cureus.21075

**Published:** 2022-01-10

**Authors:** Andrew Nguyen, Theodore Quan, Chapman Wei, Chaplin Wei, Michael-Alexander Malahias

**Affiliations:** 1 Department of Orthopaedic Surgery, Yale University, New Haven, USA; 2 Department of Orthopaedic Surgery, George Washington University School of Medicine and Health Sciences, Washington, USA; 3 Department of Orthopaedics and Traumatology, Clinica Ars Medica, Gravesano, CHE

**Keywords:** asia, journals, publications, korea, japan, china, orthopaedic

## Abstract

Introduction

Over the past two decades, Asia has experienced the rise and integration of Western medicine and digital health in its field of medicine. In this study, we investigated the trends in orthopaedic publications from three Asian countries: China, Japan, and Korea.

Methods

PubMed was used to measure the number of publications from China, Japan, and Korea in the past 21 years, from 1998 to 2020. The average percentage change in publications during this 21-year time period was analyzed using descriptive statistics. The average annual change in the number of publications from each country was also determined. One-way analysis of variance and two-group t-tests were utilized for statistical analyses with a p-value of <0.05 as the cut-off value for statistical significance.

Results

From years 1998 to 2020, there was a mean 35.5% ± 70.7% annual increase in the number of total publications from China, in comparison to a 5.1% ± 14.0% annual increase from Japan (p = 0.005) and a 27.3% ± 40.0% annual increase from Korea (p = 0.586).

Conclusion

For the past two decades, there has been a strong positive trend regarding the total number of orthopaedic publications from China. This finding might be related in part to an increased integration of Western medicine and the use of digital medicine, which followed a similar trend during the time period we analyzed. Korea and Japan also exhibited a positive trend in orthopaedic publications, which may be indicative of an improving educational system and greater general support for research.

## Introduction

Over the past 20 years, Asian countries have been integrating Western medicine practices and technologies into their clinical practice [1]. These practices have not only altered diagnoses and treatments but have also made waves in the capacities of education and research in Asia. These achievements were largely contributed to by the socioeconomic changes that have allowed an open policy for the international community to engage in collaborative research [2].

With regards to orthopaedic surgery, the growth in the number of peer-reviewed orthopaedic journals and the increased generalized importance of obtaining publications have led to the increase of articles in peer-reviewed orthopaedic journals over time [3]. Many institutions are collaborating with one another to exchange ideas and to increase their publication count [4]. Another reason for the increase in publications in orthopaedic surgery over the years is the increased awareness of bone and joint diseases [5]. Countries, such as China, have provided monetary rewards for each article accepted into a journal, which may have resulted in the increase in publications in these countries in the past ten years [6]. Of publications from eastern Asian countries, China quickly rose to become one of the largest contributors to orthopaedic surgery literature [7]. Interestingly, in February 2020, China instated a law prohibiting cash incentives for publishing articles [8]. Given this new law instated by the Chinese government, it may have a significant impact on the level of orthopaedic publications coming from Asia. Therefore, it is reasonable to assess and track the trend of publications from China up until 2020 and compare it with other Asian countries.

In this study, we sought to assess the contributions that Asian countries have provided to the field of orthopaedics. We analyzed the trend in total publications of six major orthopaedic journals from China and compared this to Korea and Japan. We suspect that Asia’s increased acceptance of Western medicine and developments in digital health are associated with a positive trend regarding publications in major orthopaedic journals.

## Materials and methods

The PubMed advanced search builder was used to measure the number of publications in six major orthopaedic journals that came from three countries: China, Japan, and Korea, in the past 21 years, from 1998 to 2020. The six major orthopaedic journals that were selected were: Journal of Arthroplasty, The Bone and Joint Journal, British Journal of Sports Medicine, American Journal of Sports Medicine, Journal of Bone and Mineral Research, and Journal of Shoulder and Elbow Surgery. These journals were selected and analyzed based on their total number of citations and impact factors according to the SCImago Journal Rank [9,10]. To measure the number of publications from the three countries, we searched for publications that reported their country as “China,” “Japan,” or “Korea” in the affiliation and author information categories.

Statistical analysis

The results from each year for each country were directly downloaded from PubMed. The average percent change in publications during this 21-year time period was analyzed using descriptive statistics. The average annual change in the number of publications from each country was also ascertained. One-way analysis of variance and two-group t-tests were utilized to make comparisons between the number of publications from China, Japan, and Korea where appropriate. A p-value of <0.05 was statistically significant.

## Results

During the study period from 1998 to 2020, there was a total of 1,227 publications from China in the six major orthopaedic journals. A total of 2,278 publications from Japan and 1,490 publications from Korea were seen in the six journals we analyzed (Figure 1). A significant difference was seen between the total number of publications from China, Japan, and Korea by year since 1998 [F (2,66) = 4.81; p = 0.011]. During this 21-year study period, there was a mean 35.5% ± 70.7% annual increase in the number of publications from China, in comparison to a 5.1% ± 14.0% annual increase from Japan (p = 0.005) and a 27.3% ± 40.0% annual increase from Korea (p = 0.586).

In the year of 1998, there were a total of three publications from China in the six major orthopaedic journals we analyzed. In the year of 2020, the total number of publications in these six journals from China was 208, which was the highest number out of all of the years in the study period, representing a 6,833% increase. Our results show that there were more publications from China in the six major orthopaedic journals in just the year 2020 (208 publications) than there were in the 13 years from 1998 to 2010 (151 publications) (Figure 2). In the year 2020, there were 56 publications in the Journal of Arthroplasty, 22 publications in The Bone and Joint Journal, nine publications in the British Journal of Sports Medicine, 41 publications in the American Journal of Sports Medicine, 40 publications in the Journal of Bone and Mineral Research, and 30 publications in the Journal of Shoulder and Elbow Surgery (Figure 2).

**Figure 1:** Comparison of the total number of publications from China, Japan, and Korea in the six major orthopaedic journals from the years 1998 to 2020.

**Figure 2:** Comparison of the number of publications from China in the six major orthopaedic journals from the years 1998 to 2020.

## Discussion

Our study shows an increasing trend in the number of publications from Asian countries in the major orthopaedic journals. In February 2020, China instated a new law prohibiting cash incentives for publishing articles to stop authors from inappropriately publishing and citing [8]. While it was reasonable to presume that the number of publications from China may have had an impact on overall publications arising from Asia in the top six orthopaedic journals after this policy, the number of publications continued to increase in the year 2020. This indicates that researchers continue to publish articles despite not receiving any cash incentives.

The results of our paper were consistent with previous studies [7]. From 1998 to 2020, China demonstrated a positive trend in orthopaedic research. In 2019 alone, the number of Science Citation Index (SCI)-cited publications for orthopaedic research from China reached 1,487 papers, accounting for 11.4% of SCI papers in the field of orthopaedics worldwide [11]. The growth of the country’s scientific contributions could be attributed to the support of the National Natural Science Foundation of China (NSFC). In the last decade, 1,938 papers were published with financial and grant support from the NSFC for orthopaedic research, accounting for 20.8% of publications from China [11]. Adequate support-in both funding and policy-has not only rapidly increased the country’s output of research in the field, but has also promoted the growth of young talent on the orthopaedic frontier through organizational support like the Young Scientists Fund [11].

The annual increase in the total number of orthopaedic publications in Korea showed a considerable evolution in their scientific research in the past twenty years. At the start of the analyzed time period, Korea developed the Visible Korean Human (VKH), being one of the few countries to make contributions to visible human research alongside the US and China [12]. In addition to contributions from their researchers and medical practitioners, the expansion of scientific publications can be attributed to the country’s greater emphasis on academic research and global involvement. The Korean orthopaedic community has pushed to improve research performance by similarly providing research awards and funding, and the Korean government has worked to foster international joint research and networking activities between researchers at the world’s top universities and research institutes [13]. These initiatives appear to be fruitful as there were many years in the analyzed time period where Korea had the highest number of orthopaedic articles published when adjusted by population and gross domestic product (GDP) [14,15]. This rapid expansion may be indicative of an improving Korean educational system and increased funding and support for researchers in the orthopaedic field.

On the other hand, our study showed that the annual increase in the total number of orthopaedic publications in Japan was not as large as that in China or Korea. This is not surprising as the Japanese government has also decreased the amount of funding available for research in the country [16]. Their shift in government policy in forcing academic institutions to become more financially independent has made them less financially incentivized to support research projects while being more incentivized for better clinical management. Additionally, this may lead to long-term obstacles in maintaining publications in orthopaedic literature as there are fewer mechanisms to secure funding for young scientists. Future government policy changes and opportunities may be needed to provide financial security to passionate young scientists in Japan to continue research in the orthopaedic field.

The observations from this study suggest that the new law instated by China prohibiting cash incentives for publishing articles has not affected the number of publications coming from China in 2020, as the numbers continue to rise. There may be a few reasons for these observations. There may be a lag time between publications being indexed on PubMed. Additionally, studies have shown that the increased international collaborations are correlated with publications in higher impact journals [17]. Seeing that there is increased international collaboration between Chinese and other researchers in the orthopaedic field, it may not be surprising to observe these increased publications from China in the most impactful orthopaedic journals [7]. Future studies should examine the number of publications from China in 2021 to assess the more long-term impact effect of this new policy.

This study has several limitations. The PubMed advanced search builder was dependent on publications reporting their country as “China,” “Japan,” or “Korea” under affiliation in the details in order to be counted as a publication from one of the countries. Therefore, the true yield of publications from these countries may be greater than what our results showed. Moreover, the predominance of the English language may be a reason why there may be a greater number of articles in these journals than our results suggest, since writing in a foreign language may be a hindrance to a country’s researchers. Additionally, this study did not provide metrics for original studies with high impact. The quantity of publications alone may not accurately reflect the true impact, especially if papers were published as follow-up studies or had relatively low citations.

## Conclusions

For the past two decades, there has been a strong positive trend regarding the total number of publications from Asian countries, specifically China, in orthopaedic journals. This finding might be related in part to an increased integration of Western medicine, increased funding for orthopaedic research, and increased international collaboration on studies. Korea also exhibited a similar positive trend in orthopaedic publications, whereas Japan only experienced a slight increase in the number of publications during the time period examined in the study.
